The article "Comparison of Biofilm and Attachment Mechanisms of a Phytopathological and Clinical Isolate of Klebsiella pneumoniae Subsp. pneumoniae" was published in 2013. Journal: ScientificWorldJournal.

# Comparison of Biofilm and Attachment Mechanisms of a Phytopathological and Clinical Isolate of* Klebsiella pneumoniae* Subsp. *pneumoniae*

**DOI:** 10.1155/2013/925375

**Published:** 2013-10-10

**Authors:** Adriana Marcia Nicolau Korres, Gloria Maria de Farias V. Aquije, David S. Buss, Jose Aires Ventura, Patricia Machado Bueno Fernandes, Antonio Alberto Ribeiro Fernandes

**Affiliations:** ^1^Núcleo de Biotecnologia, Universidade Federal do Espírito Santo, Avenida Marechal Campos 1468, 29040-090 Vitória, ES, Brazil; ^2^Instituto Federal de Educação, Ciência e Tecnologia do Espírito Santo, Campus Vitória, Avenida Vitória 1729, 29040-780 Vitória, ES, Brazil; ^3^Instituto Federal de Educação, Ciência e Tecnologia do Espírito Santo, Campus Vila Velha, Avenida Ministro Salgado Filho S/N**º**, 29106-010 Vila Velha, ES, Brazil; ^4^Instituto Capixaba de Pesquisa, Assistência Técnica e Extensão Rural do Espírito Santo, INCAPER, Rua Afonso Sarlo 160, 29052-010 Vitória, ES, Brazil

## Abstract

Some bacterial species can colonize humans and plants. It is almost impossible to prevent the contact of clinically pathogenic bacteria with food crops, and if they can persist there, they can reenter the human food chain and cause disease. On the leaf surface, microorganisms are exposed to a number of stress factors. It is unclear how they survive in such different environments. By increasing adhesion to diverse substrates, minimizing environmental differences, and providing protection against defence mechanisms, biofilms could provide part of the answer. *Klebsiella pneumoniae* subsp. *pneumoniae* is clinically important and also associated with fruit diseases, such as “pineapple fruit collapse.” We aimed to characterize biofilm formation and adhesion mechanisms of this species isolated from pineapple in comparison with a clinical isolate. No differences were found between the two isolates quantitatively or qualitatively. Both tested positive for capsule formation and were hydrophobic, but neither produced adherence fibres, which might account for their relatively weak adhesion compared to the positive control *Staphylococcus epidermidis* ATCC 35984. Both produced biofilms on glass and polystyrene, more consistently at 40°C than 35°C, confirmed by atomic force and high-vacuum scanning electron microscopy. Biofilm formation was maintained in an acidic environment, which may be relevant phytopathologically.

## 1. Introduction

Bacteria are unicellular microorganisms that live in many different environments but rarely as individual cells. Some species form an organized exopolysaccharide (EPS) structure around the cell wall, known as a capsule [1]. On a larger scale, clusters of bacteria sometimes form organized communities known as biofilms. Biofilm may be defined as an assemblage of microorganisms adherent to each other and/or to a surface and embedded in a matrix of exopolysaccharides (EPS) [2, 3].

The article "Comparison of Biofilm and Attachment Mechanisms of a Phytopathological and Clinical Isolate of Klebsiella pneumoniae Subsp. pneumoniae" was published in 2013. Journal: ScientificWorldJournal.

Bacterial adhesion and biofilm formation are very important concepts in the area of bacterial disease and control. Not only do they aid colonisation but also often provide a degree of protection against outside stresses [4]. However, the formation and structure of biofilm communities depend on a wide variety of parameters, including species, temperature, pH, and the presence of salts [2].

Various bacterial species have been found to grow on both plant and human tissues. *Klebsiella pneumoniae* subsp. *pneumoniae* has received much attention due to an association with human and animal diseases [5, 6]. Additionally, it not only has been isolated from plants including spinach [7] and rice [8] but also has recently been implicated in a disease of pineapple (pineapple fruit collapse) [9]. It is unclear how one species could be so successful on such different substrates as fruit and human tissue that it could cause disease symptoms in both. However, biofilm formation is known to be one mechanism of clinical pathogenicity of this species [10].

We proposed to investigate the adhesion and biofilm capacity of two different isolates of the important bacterial species *K. pneumoniae* subsp. *pneumoniae*, isolated from humans and pineapples.

## 2. Materials and Methods

### 2.1. Microorganisms

The bacterial isolate, *Klebsiella pneumoniae* subsp. *pneumoniae*, was obtained from pineapple fruit diagnosed with pineapple fruit collapse and identified by biochemical and physiological tests, optimal growth temperatures, partial genetic sequencing of 16S rDNA [11, 12], and comparison with the type strain. A multidrug susceptible, clinical isolate of *K. pneumoniae* subsp. *pneumoniae,* known to form slime in plate culture, was obtained by courtesy of the Marcos Daniel Clinical Laboratory (Vitória, Brazil). *Staphylococcus epidermidis* ATCC 35984 and *S. epidermidis* ATCC 12228, positive and negative for biofilm formation, respectively, were used as controls. Bacterial isolates were maintained in slant tubes of nutrient agar at 4°C.

### 2.2. Biofilm Formation in Different Surfaces

Tests for biofilm formation were performed on three different materials: glass, polyester strip, and polystyrene. Glass tubes were filled with 5 mL of tryptone-soy broth (TSB) (1.7% peptone casein; 0.3% soy peptone; 0.25% glucose; 0.5% NaCl; and 0.25% K_2_HPO_4_) at two pH values (4.5 and 7.0). Broth was inoculated with 100 *μ*L of a suspension of 10^7^ CFU·mL^−1^ of each bacterial isolate. Tubes were incubated at 35°C or 40°C for 24 h. The culture was discarded and the tube washed twice with sterile distilled water. Tubes were incubated with 0.1% safranin for 1 min. Safranin was then discarded, tubes were air-dried upside down overnight, and adherence of safranin to the inner surface of the tube was assessed visually and classified as absent (0); weak (+); moderate (++); or strong (+++) [13]. Experiments were repeated three times in triplicate.

The article "Comparison of Biofilm and Attachment Mechanisms of a Phytopathological and Clinical Isolate of Klebsiella pneumoniae Subsp. pneumoniae" was published in 2013. Journal: ScientificWorldJournal.

The polystyrene adhesion test was performed using a microplate of 96 wells [14]. Aliquots of 180 *μ*L of TSB broth and 20 *μ*L of bacterial suspension (10^7^ CFU·mL^−1^) of bacterial isolate were added to each well, and TSB broth alone was used as negative control. All sets were incubated at 35 or 40°C for 24 h in one of two pH values (4.5 and 7.0). Media were removed from the microplate by inversion, wells were gently washed with sterile distilled water, and cells adhered to the microplate were stained with 200 *μ*L of violet crystal solution (0.1%) for 30 min. The dye was discarded, and microplates dried at 40°C for 15 min. Biofilm was quantified by adding 200 *μ*L of 95% of ethanol to each well and the OD was measured at 595 nm using Elisa reader (Thermo Plate, model TP NM, Brazil) after the adjustment to zero of the negative control. Strains were considered as efficient in biofilm formation when absorbance at 595 nm was equal or the greater than 0.15 [15].

Biofilm formation was also investigated by the colony diameter test [16]. Bacterial isolate was inoculated in the center of a Petri dish containing semisolid TSB media (0.5% agar). Plates were incubated at 35 and 40°C and the diameter of the colony was measured after 5 days. The colony diameters of bacterial isolate and the negative control, *S. epidermidis* ATCC 12228, were compared, and if greater by 30% or more, the isolate was considered positive.

### 2.3. Capsule Presence by Light Microscopy

Capsule formation was assessed by the Congo red method [17]. The isolates were incubated in TSB broth at 35°C for 24 h. After this period, 2 drops of the cell suspension were mixed with 2 drops of 0.5% Congo red solution on a glass slide, and the mixture was smeared and air-dried. The material was stained with Maneval solution (1 min.), washed with distilled water, and air dried. Slides were observed under light microscope (Leica, model DMLS, Leica Microsystems, Germany) using oil immersion lens. A nonstained region around central red bacterial cells on a blue background indicated the presence of a capsule.

### 2.4. Adhesion Fiber Formation

Ability to produce adherence fibers (curli) was evaluated using a previously published protocol [18]. Plates of diluted nutrient broth (1 : 10) with 1.5% agar, Congo red (40 mg·L^−1^) and Coomassie blue (20 mg·L^−1^), were inoculated by streaking the colonies and incubated at 25°C for 48 h. Dark red or black colonies were indicative of adhesion fibers while white or pink colonies were indicative that fibers were not produced.

The article "Comparison of Biofilm and Attachment Mechanisms of a Phytopathological and Clinical Isolate of Klebsiella pneumoniae Subsp. pneumoniae" was published in 2013. Journal: ScientificWorldJournal.

### 2.5. Bacterial Hydrophobicity

Bacterial hydrophobicity was assayed by the ammonium sulfate method. Bacterial suspension (15 *μ*L) was combined with different concentrations of ammonium sulfate (0.5 M; 1 M; 1.5 M; 2 M; 2.5 M; and 3 M) (15 *μ*L) on a glass slide. The suspension was gently mixed and observed for aggregate formation for 2 min. Agglutination in salt concentrations of less than 1.0 M indicated surface hydrophobicity. Conversely, surface hydrophilicity was indicated by the agglutination of bacteria in high salt concentrations, from 2.0 to 4.0 M [19].

### 2.6. Sample Preparation for High-Vacuum Scanning Electron Microscopy (SEM) and Atomic Force Microscopy (AFM)

Biofilm formation on glass and polyester strips was also monitored visually by high-vacuum scanning electron microscopy (SEM) and atomic force microscopy (AFM). Bacterial isolate was inoculated in glass tubes with TSB as described above, and a 1 cm length dentistry polyester strip or glass coverslip was added to be settled on by the cells for microscopy experiments. Microorganisms were incubated for 20 h at 35°C. After this time, glass and polyester strips were removed from each tube, washed three times with sterile saline (0.9% NaCl), placed in sterile Petri dishes with cheesecloth, and air dried at room temperature [20].

For SEM, each sample was mounted on aluminum stubs and sputter-coated with 20 nm gold (Bal-Tec Sputter Coater SCD-050, Capovani Brothers Inc., Scotia, USA). Samples were observed using a Shimadzu SSX 550 high-vacuum scanning electron microscope (Shimadzu, Kyoto, Japan) operated at 20.0 kV.

For AFM, samples were observed using a Shimadzu SPM-9600 series Microscope (Shimatzu, Kyoto, Japan). Si_3_N_4_ cantilever tips (model OMCL-TR, Olympus, Tokyo, Japan) with a nominal constant of 32 N·m^−1^ and resonance frequency of *≈*300 kHz were used with scan rates of 0.3–1.0 Hz and scan size of 2,000–10,000 nm and imaging analysis were performed with the accompanying software.

### 2.7. Statistical Analysis

All experiments were conducted in triplicate, and repeated three times. Statistical analysis was performed by ANOVA using Multistat software by comparing the mean values by Tukey test with 5% probability [21].

## 3. Results

### 3.1. Biofilm Formation Assessment by Routine Laboratory Tests

Colony diameter tests showed that both *Klebsiella* isolates were positive for biofilm formation. Colonies of *K. pneumoniae* subsp. *pneumoniae* isolated from pineapple fruit and the clinical isolate were 152.9% and 135.3% larger, respectively, compared to negative control *S. epidermidis *ATCC 12228. The *Klebsiella* isolates were both significantly different to the control (*P* < 0.001), but not to each other (*P* > 0.05).

The article "Comparison of Biofilm and Attachment Mechanisms of a Phytopathological and Clinical Isolate of Klebsiella pneumoniae Subsp. pneumoniae" was published in 2013. Journal: ScientificWorldJournal.

*K. pneumoniae* subsp. *pneumoniae* isolated from pineapple fruit and the clinical isolate were positive for adherence to the inner surface of glass tubes and on polystyrene microtiter plates as was the positive control *S. epidermidis* ATCC 35984. Microtiter plate tests performed with both *Klebsiella* isolates demonstrated low OD values (0.130–0.212) compared to the positive control *S. epidermidis* ATCC 35984 (1.525), indicating the presence of a biofilm but at a relatively low level.

*Klebsiella* isolates formed a more consistent biofilm at 40°C than 35°C as measured by both glass adhesion and polystyrene microtiter plate assays (Table 1). There was no difference between the two *Klebsiella* isolates. Biofilm formation by both was greater than *S. epidermidis* ATCC 35984 at pH 4.5 but considerably less at pH 7.0.

### 3.2. Capsule and Adhesion Fimbriae Formation

*K. pneumoniae* subsp. *pneumoniae* isolated from pineapple fruit and the clinical isolate were both able to form capsules as shown by the Congo red test as was the positive control *S. epidermidis* ATCC 35984. However, neither of the *K. pneumoniae* subsp. *pneumoniae* isolates was able to produce adhesion fibers (curli), in contrast to *S. epidermidis* ATCC 35984.

### 3.3. Hydrophobicity

Both *K. pneumoniae* subsp. *pneumoniae* isolates demonstrated surface hydrophobicity in aggregation tests in different concentrations of ammonium sulfate, aggregating in concentrations >3.0 M. This was higher than the positive control, *S. epidermidis* ATCC 35984, which aggregated in concentrations >2.0 M.

### 3.4. Atomic Force Microscopy (AFM) and High-Vacuum Scanning Electron Microscopy (SEM)

*In situ* biofilm monitoring by high-vacuum scanning electron (Figures 1(a) and 1(b)) and atomic force microscopy (Figures 1(c) and 1(d)) showed that *K. pneumoniae* subsp. *pneumoniae* isolated from pineapple was able to form a biofilm on the surface of glass (Figures 1(a) and 1(c)) and polyester (Figures 1(b) and 1(d)).

In AFM plan view, EPS was clearly visible as cloudy areas around the cells (Figures 2(a) and 2(b)). Topographic profiles indicated that biofilm height on glass and polyester was similar (Figures 1(c), 1(d) and Figure 2); the average height of biofilm on polyester was 85.21% of the average obtained on glass. The profile of cells on glass (Figure 2(c)) was smoother whilst divisions between cells were more evident on polyester (Figure 2(d)).

The article "Comparison of Biofilm and Attachment Mechanisms of a Phytopathological and Clinical Isolate of Klebsiella pneumoniae Subsp. pneumoniae" was published in 2013. Journal: ScientificWorldJournal.

## 4. Discussion

Tests performed on *K. pneumoniae* subsp. *pneumoniae* isolated from both pineapple and human tissue, for adhesion to polystyrene and glass and comparative colony diameter, showed that these isolates are able to form biofilms. However, results suggested a lower level of biofilm formation compared to the positive control *S. epidermidis* ATCC 35984, and Congo red tests indicated that the *K. pneumoniae* subsp. *pneumoniae* isolates did not form adhesion fibers (curli). In hydrophobicity tests, the isolates were hydrophilic compared to *S. epidermidis* ATCC 35984. Together these results explain the relatively low adhesion to polystyrene microtiter plates [18, 22].

We found that in every respect the biofilm and surface characteristics of the two *K. pneumoniae* subsp. *pneumoniae* isolates were identical despite their very different origins. Both isolates of *Klebsiella* formed a consistent biofilm in both acidic (pH 4.5) and neutral (pH 7.0) environments whilst *S. epidermidis* ATCC 35984 only produced biofilm at pH 7.0. In a phytopathological context, biofilms may help bacteria survive in the highly acidic pineapple environment as the nature of the gel-like structure prevents rapid diffusion of ions and allows considerable pH gradients to develop within the matrix [23]. In contrast, it has been suggested that alkaline environments are inhibitory to *K. pneumoniae* so that the toxicity of various bioactive glasses to this species may be partly due to the release of ions in aqueous solutions, and thus an increase in pH [24].

Acidity, temperature, and ion concentration have all been shown to influence biofilm formation by microorganisms in different conditions [25]. The isolates tested here were also affected by temperature. Both *Klebsiella* isolates and *S. epidermidis* ATCC 35984 formed a more consistent biofilm at 40 than at 35°C. In a similar context, the plant rhizobacteria *Pseudomonas putida* has also been reported to tolerate temperatures of 40°C by enhanced biofilm production [26].

The survival of pathogenic bacteria outside of the human host is of crucial clinical importance, and an association with plants and plant based products is becoming more apparent. For example, plant polysaccharides, increasingly used in food packaging, have been shown to be adhesion sites for the pathogens *Escherichia coli* and *Staphylococcus aureus* [27]. Additionally, it is almost impossible to prevent the contact of clinically pathogenic bacteria with food crops. They can be applied with contaminated manure or irrigation water or via wild animals [28]. If clinically pathogenic bacteria can survive on food plants they can reenter the human food chain and cause disease [29, 30]. Bacteria on the plant surface are exposed to UV light, desiccation, and, conversely, high flow from rain and irrigation and so tend not to maintain a presence for long [31, 32]. However, if they can enter plant tissues via injuries, survival is greatly improved with contamination lasting at least 3 weeks in lettuce and chives, for example [32].

The article "Comparison of Biofilm and Attachment Mechanisms of a Phytopathological and Clinical Isolate of Klebsiella pneumoniae Subsp. pneumoniae" was published in 2013. Journal: ScientificWorldJournal.

Overall, our results showed a similar profile of biofilm and adhesion characteristics between the two *K. pneumoniae* subsp. *pneumoniae* isolates despite the differences in original substrates. This suggests a flexibility in choice of mechanisms within isolates as both adjusted equally to glass and plastic after their respective tissues, which may account for the success of this species in humans and plants and for the health problems that result.

## Figures and Tables

**Figure 1:** High-vacuum scanning electron micrographs and atomic force microscopy of *K. pneumonia* subsp. *pneumoniae*. SEM ((a) and (b)) and AFM in 3D ((c) and (d)) micrographs showing cell aggregates and biofilm on glass ((a) and (c)) and polyester ((b) and (d)).

**Figure 2:** Atomic force microscopy of *K. pneumoniae* subsp. *pneumoniae*. Topographic profile of cell aggregates and biofilm on glass ((a) and (c)) and polyester ((b) and (d)). Plan view ((a) and (b)). Cell aggregate topographical profile along the lines A-B and C-D ((c) and (d)).

**Table 1:** Biofilm formation by microorganisms on glass in different pH and temperature.

Microorganisms	pH 4.5		pH 7.0	
	35°C	40°C	35°C	40°C
*K. pneumoniae* subsp. *pneumoniae* (pineapple isolate)	+*	++	+	++
*K. pneumoniae* subsp. *pneumoniae* (clinical isolate)	+	++	+	++
*S. epidermidis* ATCC 35984	0	0	++	+++

*Absent (0); weak (+); moderate (++); or strong (+++), Stepanović et al., 2000 [13].
